This article has been retracted.

# Exosome: Function and Application in Inflammatory Bone Diseases

**DOI:** 10.1155/2021/6324912

**Published:** 2021-08-31

**Authors:** Yingkun Hu, Yi Wang, Tianhong Chen, Zhuowen Hao, Lin Cai, Jingfeng Li

**Affiliations:** Department of Orthopedics, Zhongnan Hospital of Wuhan University, Wuhan, China

## Abstract

In the skeletal system, inflammation is closely associated with many skeletal disorders, including periprosthetic osteolysis (bone loss around orthopedic implants), osteoporosis, and rheumatoid arthritis. These diseases, referred to as inflammatory bone diseases, are caused by various oxidative stress factors in the body, resulting in long-term chronic inflammatory processes and eventually causing disturbances in bone metabolism, increased osteoclast activity, and decreased osteoblast activity, thereby leading to osteolysis. Inflammatory bone diseases caused by nonbacterial factors include inflammation- and bone resorption-related processes. A growing number of studies show that exosomes play an essential role in developing and progressing inflammatory bone diseases. Mechanistically, exosomes are involved in the onset and progression of inflammatory bone disease and promote inflammatory osteolysis, but specific types of exosomes are also involved in inhibiting this process. Exosomal regulation of the NF-*κ*B signaling pathway affects macrophage polarization and regulates inflammatory responses. The inflammatory response further causes alterations in cytokine and exosome secretion. These signals regulate osteoclast differentiation through the receptor activator of the nuclear factor-kappaB ligand pathway and affect osteoblast activity through the Wnt pathway and the transcription factor Runx2, thereby influencing bone metabolism. Overall, enhanced bone resorption dominates the overall mechanism, and over time, this imbalance leads to chronic osteolysis. Understanding the role of exosomes may provide new perspectives on their influence on bone metabolism in inflammatory bone diseases. At the same time, exosomes have a promising future in diagnosing and treating inflammatory bone disease due to their unique properties.

## 1. Introduction

Bone homeostasis is a balance of osteoblasts and osteoclasts constantly acting on the bone to renew the body's bone mass. Chronic inflammation caused by various stressors can to disrupt this delicate balance between osteoblasts and osteoclasts by secreting various inflammatory factors, such as tumor necrosis factor-*α* (TNF-*α*), interleukin-1 (IL-1), interleukin-6 (IL-6), and prostaglandin E2 (PGE2), leading to disturbances in bone metabolism [1]. These osteolytic lesions caused by chronic aseptic inflammation include aseptic loosening of the prosthesis [2], osteoporosis [3, 4], and rheumatoid arthritis [5]. Aseptic loosening around the prosthesis is an outstanding representative of these disorders.

Exosomes, as transmitters of intercellular information, may be an emerging target for our exploration of the pathogenesis of inflammatory bone diseases and their therapeutic targets. Extracellular vesicles include four subgroups, namely, exosomes, microparticles, apoptotic vesicles, and cancer vesicles [10]. The current research hotspot is the subgroup of exosomes. Exosomes are disc-shaped vesicles that contain polysaccharides, lipids, metabolites, RNA (microRNA and lncRNAs), DNA, and specific proteins [11]. With a diameter of 40–100 nm, these tiny vesicles can act as signaling molecules to other cells, thereby altering the function of other cells [12]. These findings have inspired a number of studies on exosomes. Exosomes serve as an essential mediator of intercellular communication, altering the phenotype of target cells by delivering cargo into the cytoplasm. Given the selective loading of cargo, cargo composition in exosomes may differ from the tissue or cells from which they originate [13]. As in other cell types, macrophages deliver inflammatory signals by extracellular vesicles. Research increasingly shows that exosomes are involved in a variety of pathological processes, including chronic inflammation [14]. Based on the function of exosomes in delivering specific proteins and nucleic acids to specific target cells, it is reasonable to assume that exosomes could also play an essential role in intercellular communication in inflammatory bone diseases. Macrophage function is closely related to inflammation that is closely related to bone metabolism. Reversing inflammatory osteolysis by designing the effects of different types of exosomes on macrophage function and bone metabolism, and ultimately cell-free therapy, is challenging, which will also provide a new perspective for researchers. A better understanding of the pathogenesis of inflammatory bone disease has important implications for the design of novel therapeutics for inflammatory bone disease. In this comprehensive review, we highlight the effect of exosomes on inflammatory bone disease through their roles in inflammation and bone metabolism. Enhanced osteoclast activity and diminished osteoblast activity are the two main aspects of bone metabolism disorders in inflammatory bone diseases. However, the body also self-regulates and produces protective exosomes to counteract this process. Finally, we discuss the possible applications of exosomes in inflammatory bone diseases in clinical diagnosis and treatment.

## 2. Overview of Exosomes

Exosomes are extracellular vesicles from the endosomal pathway in the nanometer diameter range that can be secreted by most cells under physiological or pathological conditions by cytosolic exocytosis [15]. Exosomes are widely found in various body fluids of living organisms, such as blood, urine, saliva, ascites, and bile. The secretory pathway of exosomes has been extensively studied since its discovery, and exosomes from different cells have similar effects to their parent cells. Exosomes are involved in many physiological and pathological processes, including tissue damage and repair responses, by coordinating the communication between different cell types. They act as vectors between different cell types that transfer nucleic acids, proteins, or lipids to target cells, causing changes in the phenotype and function of the target cells [16]. More than 41,860 proteins, 7,540 RNAs, and 1,116 lipid molecules have been identified in exosomes [17]. The formation of exosomes involves the following steps: first, inward budding of endosomal membranes to generate multivesicular bodies (MVBs); then, MVBs fuse with the plasma membrane and release their luminal vesicles to form exosomes [18]. Exosomes can travel throughout the body via the circulatory system and cross the blood-brain barrier and other tissues to be taken up by target cells (Figure 1). Extracellularly, signals are delivered from exosomes to recipient cells in three ways: receptor-ligand binding, membrane fusion, or phagocytosis [19]. Exosome secretion occurs naturally in organisms, and stress and inflammatory signals can regulate the processes involved [20].

Exosomes may play an essential role in sterile inflammation, including prosthesis loosening, because they can modulate immunity by transmitting inflammatory signals and regulating macrophage differentiation [21]. A growing number of studies emphasize the role of exosomes in inflammation-associated intercellular communication. Currently, only a few studies have been conducted on exosomes associated with aseptic loosening compared with other aseptic inflammatory conditions of the bone. The limited studies may be because experimental models of aseptic loosening are more complex and challenging to establish than those of other disease pathogenesis. However, it may share similar signaling cascades with diseases, such as rheumatoid arthritis and osteoarthritis, although such diseases are mediated by different triggers. Some of the pathogenic processes associated with the development of inflammatory bone diseases in exosomes include the delivery of miRNAs, lncRNAs, inflammatory cytokines, chemokines, proteases, and other proteins; activation of macrophages; activation of Toll-like receptors; intercellular communication; and degradation of the extracellular matrix.

## 3. Exosomes and Macrophage Polarization

Macrophage polarization is closely associated with inflammatory bone disease. Excessive numbers of macrophages or M1 polarization can induce delayed bone healing and chronic inflammation. Chronic inflammation leads to the production of various inflammatory factors that cause progressive osteolysis, as well as inhibit bone formation. Macrophages, as regulators of inflammation, are central to the pathogenesis of inflammatory bone diseases due to aseptic inflammation. Macrophages are important coordinators of immune activity and homeostasis in the body and are involved in the elimination of foreign substances, relief of inflammation, and tissue repair. At present, macrophages are recognized to play an important role in the etiology of inflammatory bone diseases. Macrophages in areas of inflammatory tissue are derived from monocytes in the bloodstream. Activated macrophages can be categorized into the M1 phenotype (classically activated macrophage phenotype) and the M2 phenotype (alternative activated macrophage phenotype) [22]. In the presence of interferon *γ* (IFN-*γ*) and lipopolysaccharide (LPS), macrophages polarize toward the M1 phenotype. Nevertheless, in the presence of interleukin-4 (IL-4), another well-known cytokine produced by T cells, macrophages polarize to the M2 phenotype. Macrophage polarization induced by various stressors, such as abrasive debris in aseptic loosening, favors the M1 phenotype. M1 phenotype macrophages play a defensive role when interacting with biological materials. They perform phagocytic functions to remove pathogens and debris from injury sites and perform proinflammatory functions by secreting TNF-*α*, IL-1, and IL-6 [23]. M2 phenotype macrophages exert anti-inflammatory effects and secrete interleukin-10 (IL-10) [24]. The dynamic balance between M1-like and M2-like macrophages strictly controls the outcome of the disease. Macrophage polarization toward the M1 phenotype is one of the most important manifestations in the development of aseptic bone inflammation. Nuclear factor-*κ*B (NF-*κ*B) is a key transcription factor in macrophages that regulates macrophage polarization. An increasing number of studies have found that exosomes can alter the polarization phenotype of macrophages by stimulating the NF-*κ*B signaling pathway and a variety of other pathways (Figure 2).

### 3.1. Exosomes Activate Toll-Like Receptors

Innate immune cells use their pattern recognition receptors to detect pathogen-associated molecular patterns and damage-associated molecular patterns, which play a decisive role in host defense against invading pathogens [8]. As a characteristic representative of pattern recognition receptors, the Toll-like receptor (TLR) is known to identify endogenous and infectious stress that triggers inflammation and aids in adaptive immune responses. It is intriguing that exosomes can also activate Toll-like receptors to trigger inflammatory responses. Plasma exosomes from patients with rheumatoid arthritis can activate TLR4, and this activation mechanism is similar to that of TLR4 activation by LPS [25]. Further studies showed that oxidized phospholipids on exosome membranes are responsible for the stimulation of TLR-4 [25]. TLR4 can recruit MyD88 when it is activated. The binding of TLR4 and MyD88 phosphorylates IRAK4, which in turn phosphorylates IRAK1. The tight packing of IRAKs activates their potential kinase activity, driving autophosphorylation and subsequent recruitment of the E3 ubiquitin ligase TRAF6. TRAF6 activates the kinase TAK1, which stimulates I*κ*B kinase- (IKK-) mediated NF-*κ*B and mitogen-activated protein kinase- (MAPK-) mediated AP-1 transcriptional responses [26]. In a nutshell, the MyD88-dependent pathway leads to activation of NF-*κ*B and activator protein-1 (AP-1) that promote the secretion of proinflammatory cytokines, such as TNF-*α*, IL-1, and IL-12. Exosomes act as an endogenous danger signal induced by oxidative stress and play a vital role in the onset and development of inflammatory bone diseases.

The process of aseptic loosening also involves the activation of Toll-like receptors. For example, TLR1/TLR2 heterodimer can be activated by UHMWPE, while TLR4 can be activated by cobalt or nickel ions [27, 28]. However, no further studies have been done to investigate whether exosomes are involved in this process in aseptic loosening. Recent studies have found that TLR can be transmitted between immune cells via exosomes and can increase the responsiveness of recipient cells to LPS [29]. These findings show that exosomes play an essential role in the activation of Toll-like receptors. Whether exosomes have other roles on Toll-like receptor activation in inflammatory bone diseases, such as whether exosomes can activate other subtypes of Toll-like receptors and the conditions of activation, remains to be further explored.

### 3.2. Exosomes Contain a Variety of Inflammatory Cytokines

Macrophage-derived exosomes represent a significant fraction of the exosomal component of the blood. Several studies have found that exosomes produced by immunocytes, such as macrophages and dendritic cells, contain various proteins without N-terminal signaling peptides, including chemokines and inflammatory cytokines [30]. These exosomal components can influence the progression of inflammatory bone diseases, but their effects are not dependent on the exosome structure. In other words, these inflammatory and chemokine components are present in exosomes, are widely distributed in the body, and are involved in the process of inflammatory bone diseases. Inflammatory cytokines promote NF-*κ*B expression through activation of the NF-*κ*B signaling pathway by cytokine receptors to regulate macrophage polarization.

Exosomes isolated from patients with rheumatoid arthritis contained a membrane-bound form of tumor necrosis factor-*α*, which activates NF-*κ*B and leads to the induction of matrix metalloproteinase-1 (MMP-1) [31]. Inflammatory cytokines, such as TNF-*α* and IL-1*β*, can cause an inflammatory cascade around the prosthesis. TNF-*α* is the major anti-M2 inflammatory cytokine that impedes M2 macrophage production by acting directly on unactivated macrophages and affecting IL-13 production and AMPK phosphorylation in other cell types [32]. TNF-*α* also activates macrophages to release other inflammatory cytokines, such as IL-6 and IL-1*β*, which promote inflammatory responses. However, the membrane-bound form of TNF-*α* should be cleaved into a soluble form to promote osteoclast formation. IL-1*β*, a critical inflammatory cytokine in the inflammatory cascade response, is also secreted in exosomal form as an essential adjunct to its output [33–35]. IL-1*β* is not only released by cells during the fusion of secretory lysosomes with the plasma membrane but is also secreted by exosomes [36]. When ATP binds to P2X7R in the exosome, IL-1*β* is released from the exosome to regulate the inflammatory response [37]. IL-1*β* is considered one of the most important family members of the interleukin family with intense proinflammatory activity by stimulating the production of various proinflammatory mediators, such as cytokines, chemokines, and matrix metalloproteinases (MMPs) [38]. IL-1*β* and IL-6 act synergistically and activate each other's expression, with positive feedback leading to the continued progression of chronic inflammation. Production of monocyte chemoattractant protein-1 (MCP-1), IL-6, IL-8, and PGE2 is increased in bone marrow mesenchymal stem cells in response to IL-1 exposure [39]. The expression of IL-1*β* and TNF-*α* is driven by NF-*κ*B, and in turn, they are also potent activators of the NF-*κ*B pathway. The content of cytokines, especially chemokines, in macrophage-derived exosomes increases after LPS stimulation [40]. Similar experimental studies found elevated levels of chemokine (CC motif) ligand 3 (CCL3), also called MIP1*α* (macrophage inflammatory protein-1*α*), in exosomes secreted by macrophages after LPS treatment [41]. CCL3 acts as a chemotactic factor responsible for the recruitment of monocytes/macrophages at sites of inflammation. In prosthetic aseptic loosening, polymethylacrylate particles stimulate RAW 264.7 cell-induced MSC chemotaxis due to CCL3 as it can be blocked by CCL3 inhibitors [42]. In addition, exosomes isolated in monocytes were found to transport arachidonic acid, a precursor of the inflammatory factor PGE2, into fibroblast-like synoviocytes of patients with rheumatoid arthritis [43]. PGE2 is a paracrine factor released from mesenchymal stem cells with powerful immunomodulatory functions and upregulates IL-10 secreted by macrophages and stimulates M2 macrophage polarization to accelerate the recovery of damaged tissues [44]. However, PGE2 also promotes RANKL expression in periprosthetic fibroblasts [45].

Functionally, exosomes containing inflammatory factors resemble inflammatory cells, modulate the expression of inflammatory responses, and have an essential role in the regulation of inflammatory bone disease. However, a complete spectrum of exosome-associated inflammatory cytokines is still not available, probably due to the inability of the technology to completely distinguish conventional cytokines from those in exosomes. Therefore, the changes in the content of and the intensity of action of these inflammatory factors in exosomes of skeletal aseptic inflammation have not been well studied.

### 3.3. Exosomal Delivery of RNA Promotes Macrophage Polarization

Exosomes can transport inflammatory factors and control the expression of inflammatory factors to promote the inflammatory response. Exosomes from IL-1*β*-treated synovial fibroblasts could induce osteoarthritis-related gene expression changes in articular chondrocytes, including upregulation of MMP-3, MMP-13, IL-6, and VEGF [46]. Another prominent example is that exosomes secreted by TNF-*α*-treated monocytes and T cells can directly stimulate the secretion of inflammatory mediators IL-6 and IL-8 by fibroblast-like synoviocytes [43]. Exosomes derived from SF cells from patients with end-stage osteoarthritis promote the macrophage expression of a range of proinflammatory factors, such as IL-1*β*, IL-6, chemokines, MMP-7, and MMP-12 [47].

Several studies have further explored the mechanisms through which exosomes promote inflammatory responses. The expression levels of exosomes containing lncRNA Hotair were significantly elevated in rheumatoid arthritis sera, leading to the migration of activated macrophages [48]. This phenomenon may be attributed to lncRNA Hotair that regulates the activation of NF-*κ*B and the expression of its target genes (IL-6 and iNOS) by promoting I*κ*B*α* degradation [49]. In rheumatoid arthritis, miR-106b is highly expressed in fibroblast-derived exosomes [50]. miR-106b promotes macrophage polarization and increases osteoclast formation by activating phosphatase and tensin homolog/phosphatidylinositol 3-kinase/serine/threonine-protein kinase (PTEN/PI3K/AKT) and NF-*κ*B signaling pathways [51]. miR-106b promotes the phosphorylation of I*κ*B-*α* and p65, thereby facilitating the activation of NF-*κ*B signaling in macrophages.

As such, these inflammation-induced exosomes affect macrophage activation via NF-*κ*B signaling. These may also help to reveal the mechanism of TNF-*α*- and IL-1-induced NF-*κ*B activation. NF-*κ*B, in turn, is responsible for the transcription of many genes for proinflammatory cytokines and chemokines. These exosomes, which have a proinflammatory response, form positive feedback with inflammatory factors and promote the development and progression of inflammatory bone disease.

### 3.4. Exosomes Prevent Overactivation of the Inflammatory Response

Macrophage-derived exosomes not only promote the development of aseptic inflammation but also play a role in preventing the overactivation of the immune response. LPS-stimulated macrophages secrete exosomes carrying higher levels of three miRNAs (miRNA-21-3p, miRNA-146a, and miRNA-146b) than those of unactivated macrophages. These three miRNAs can inhibit the release of inflammatory factors from macrophages by suppressing NF-*κ*B expression and Toll-like receptor activation [52, 53]. In addition, further studies revealed that miR-21, induced by NF-*κ*B, can act as an inflammatory suppressor involved in the regulation of protective cytokines IL-4 and IL-10 [54, 55]. It may partially explain why IL-10 is elevated in patients with aseptic loosening of the prosthesis. Another study reported that macrophage-derived exosomes have high levels of miR-223 [56]. miR-223 suppresses inflammatory responses by targeting IKK*α* and inhibiting nonclassical NF-*κ*B signaling during macrophage differentiation [57, 58]. However, miR-223 can induce differentiation of monocytes to macrophages by regulating inositol phosphatase, which is essential for monocyte survival [56].

Mesenchymal stem cell-derived exosomes are the most vital force that prevents overactivation of the inflammatory response in aseptic inflammation of the bone. The anti-inflammatory effects of MSC-derived exosomes have been described in several scenarios. Several studies have shown that MSC-derived exosomes can attenuate macrophage polarization and recruitment. This finding is exemplified in work undertaken by Shen et al. [59]. They found that MSC-derived exosomes express CC motif chemokine receptor 2, which plays a crucial role in preventing macrophage accumulation and tissue damage by inhibiting its activity through binding to the proinflammatory chemokine CCL2 as a decoy receptor. CCL2, also called MCP-1, is the most critical chemokine that regulates the migration of monocytes and macrophages. Macrophages and monocytes migrate toward a slope of CCL2 via its receptor CCR2. Titanium particles lead to increased CCL2 secretion [60]. Cosenza et al. demonstrated for the first time that MSC-derived exosomes play an immunomodulatory role in inflammatory arthritis [61]. In addition, various disease models have illustrated the effect of MSC-derived exosomes on the M1/M2 polarization of macrophages. Gingival tissue-derived MSCs showed a rapid increase in exosome secretion after TNF-*α* treatment, which also enhanced CD73 exosome expression and promoted the polarization of M2 macrophages [62]. Several studies have further investigated the regulatory mechanisms through which MSC-derived exosomes affect macrophage polarization. MSC-derived miR-150-5p exosomes reduced migration and invasion of fibroblast-like synovial cells in patients with rheumatoid arthritis by targeting MMP-14 and VEGF [63]. In another study, Xu et al. found that exosomes derived from bone marrow MSCs pretreated with LPS reduced the phosphorylation level of I*κ*B, thus inhibiting the LPS-dependent NF-*κ*B signaling pathway [64]. However, they did not indicate the exosome component that caused this result. These findings may provide new ideas for the treatment of inflammatory bone diseases.

Taken together, macrophages can secrete several exosomes containing unique microRNAs that are involved in preventing the overactivation of the inflammatory response. In addition, MSC-derived exosomes may have similar effects to MSCs and are major anti-inflammatory exosomes. They can induce macrophage shift from the M1 phenotype to the M2 phenotype, inhibit proinflammatory cytokines, release anti-inflammatory cytokines, inhibit the progression of inflammatory bone diseases, and attenuate periprosthetic osteolysis. Although the inflammatory response is essential in resisting various external stresses, it is also a double-edged sword. During inflammation, exosomes released by various cells are simultaneously inhibiting the course of the inflammatory response, which may be a self-protective effect of the organism. Nevertheless, this coordination of anti-inflammatory effects does not entirely stop the progression of inflammatory bone disease. The exosomes contain goods with both proinflammatory and anti-inflammatory effects to buffer the inflammatory response of the receptor cells to an optimal magnitude of response. This simultaneous proinflammatory and anti-inflammatory mechanism results in a weak inflammatory state, which allows the disease to last for years or even decades.

## 4. Exosomes and Bone Metabolism

### 4.1. Exosomes and Bone Resorption

Osteolysis due to increased osteoclast activity is the primary pathological process in the development of inflammatory bone disease to a specific stage. The osteoclast, whose specific marker is the expression of tartrate-resistant acid phosphatase (TRAP), is the only cell type that participates in the destruction and resorption of bone tissue in living organisms. Osteoclasts are differentiated from hematopoietic stem cell-derived monocytes and macrophage lineage progenitors (progenitors of osteoclasts). Osteoblasts secrete the macrophage colony-stimulating factor (M-CSF) and act on osteoclast progenitors to promote their survival, while the receptor activator of nuclear factor-kappaB ligand (RANKL) is secreted to promote osteoclast precursor cell differentiation [65]. When RANKL binds to the receptor activator of nuclear factor-kappaB (RANK) expressed in the osteoblast precursor cells, ligand proteins, such as tumor necrosis factor receptor-associated factor-6 (TRAF6), bind to the intracellular domain of RANK. Then, kinases, such as NF-*κ*B, extracellular signal-regulated kinase (ERK), Jun N-terminal kinase (JNK), and p38 are activated [66]. Eventually, osteoclast precursor cells differentiate into osteoblasts by expressing c-Fos and nuclear factor of activated T cells (NFATc1), transcription factors of specific genes, such as tartrate-resistant acid phosphatase (TRAP), and cathepsin K, for osteoclast differentiation [67, 68]. As in inflammation, exosomes are involved in several processes, such as promoting osteolysis and inhibition of osteolysis (Figure 3).

#### 4.1.1. Exosomes Directly Promote Differentiation of Osteoclasts

Osteoclasts can take up exosomes by phagocytosis and are affected by the various cargoes carried by exosomes [69]. RANKL, a growth factor essential for osteoclast differentiation, was identified in 2015 as expressed in exosomes secreted by osteoblasts and stromal cells [70]. Isolation of RANKL-containing exosomes from mouse cranial osteoblasts was shown to stimulate the differentiation of monocytes/macrophages into osteoclasts [71]. Recent in vivo experiments have demonstrated that RANKL-containing exosomes released from osteoblasts can target osteoclasts and stimulate osteoclast formation [72]. The targeted delivery of RANKL-containing exosomes to osteoclasts may be related to the interaction of RANKL on the surface of the exosome membrane with RANK on the surface of the osteoclast precursor membrane [70]. Studies have shown that after parathyroid hormone treatment, osteoblasts secrete more RANKL-containing exosomes, causing an increase in osteoclast differentiation [73]. In another study, RANKL levels in synovial exosomes were significantly higher in patients with rheumatoid joints [74]. Exosomes likely promote osteoclast differentiation directly through RANKL transport. Nevertheless, now, RANKL levels in exosomes are not well measured in other sterile bone inflammatory conditions, such as aseptic loosening.

In addition, Li et al. found that miR-214 expression in osteoblasts was positively correlated with miR-214 levels in serum exosomes and that patients with osteoporotic fractures had higher miR-214 levels than normal subjects [75]. Further studies showed that miR-214 targeted to block PTEN expression and activated the PI3K/Akt signaling pathway, thereby enhancing osteoclast formation [76]. Exosomes containing miR-106b can also promote osteoclastogenesis by regulating the PTEN/PI3K/Akt pathway [51]. PTEN is a repressor gene of Akt and inhibits Akt activation by dephosphorylating PIP3 to antagonize the activity of PI3K. The activated PI3K/Akt pathway inhibits glycogen synthase kinase 3*β* (GSK-3*β*) through phosphorylation, and this GSK-3*β* inhibition leads to nuclear localization of NFATc1, resulting in enhanced osteoclastogenesis [77].

Exosomes can regulate osteoclast activity by promoting the expression of inflammatory factors and by direct activation of osteoclasts via transported cargo. Multiple mechanisms act together to trigger osteolysis in sterile bone inflammation.

#### 4.1.2. Exosomes Indirectly Promote Osteoclast Differentiation through Inflammatory Factors

Some specific exosomes derived from inflammatory bone diseases promote the expression of a range of inflammatory factors, including TNF-*α*, IL-1, and VEGF, which increase osteoclast activity [78, 79]. TNF-*α* promotes periprosthetic bone resorption by enhancing RANKL and M-CSF expression in osteoblasts, osteocytes, and stromal cells and enhancing the sensitivity of osteoclast precursors to RANKL [80]. This mechanism of promoting RANKL-induced osteoclast formation may be accomplished by inducing the expression of Blimp1, a transcriptional repressor that plays a critical role in the differentiation and function of a variety of cells, including osteoclasts [81]. However, in the absence of RANKL and osteoblast/stromal cells, TNF-*α* stimulates osteoclast differentiation in the presence of M-CSF [82]. Although transient exposure of bone marrow MSCs to TNF-*α* increases osteogenesis in vitro, continued stimulation with TNF-*α* leads to osteoclast activation and impaired osteoblast function. IL-1, another inflammatory factor promoted by expression in sterile bone inflammatory exosomes, enhances RANKL expression in osteoblasts and stromal cells and may directly stimulate the differentiation of osteoclast precursors through an alternate pathway (RANKL independent). This RANKL-independent osteoclast induction may be related to IL-1*α*-induced expression of microphthalmia transcription factor (MITF) in macrophages [83]. VEGF is also carried by exosomes as a cargo [84]. VEGF acts as an osteolytic agent in a paracrine manner in inflammatory bone diseases. It also plays a role in the chemotaxis and proliferation of osteoclast precursors, inducing osteoclastogenesis [85].

#### 4.1.3. Exosomes Affect the Degradation of the Extracellular Matrix

Exosomes derived from monocytes and T cells stimulated by inflammatory factors, such as TNF-*α*, induce high production of MMP-1, MMP-3, MMP-9, and MMP-13 by rheumatoid arthritis fibroblasts [86]. Matrix metalloproteinases (MMPs) are a family of 23 structurally related proteolytic enzymes, which can degrade almost all components of the extracellular matrix [87]. MMP-9 promotes bone resorption by degrading extracellular matrix macromolecules around and on the surface of bone trabeculae and mediates osteoclast adhesion and migration to resorption sites [88]. MMP-13, which breaks down proteoglycans in the extracellular matrix, such as proteoglycans and collagen, is thought to be the main protease responsible for cartilage destruction in rheumatoid arthritis [78]. Several studies demonstrated that many MMPs might lead to prosthetic loosening and osteolysis through pathological extracellular matrix degradation and periprosthetic connective tissue/bone remodeling [89–92]. Periprosthetic fibroblast-like cells express MMP-13 in response to induction of wear particles, and the increase in matrix metalloproteinases destroys the periprosthetic tissue [45]. Blocking TNF-*α* and IL-1*β* receptors does not attenuate the damaging effects of exosomes on the extracellular matrix, suggesting that the mechanism of increased matrix metalloproteinase production caused by exosomes is independent of the TNF-*α*-induced inflammatory response. Exosomes secreted by fibrous synovial cells from rheumatoid patients carry high levels of ADAMTS-5, and exosomes isolated from endothelial cells contain MMP-2, MMP-9, and MMP-14 [78]. This finding suggests that exosomes from patients with aseptic bone inflammation can break down bone tissue directly. Exosomes directly mediate the destruction of the bone matrix through matrix metalloproteinases, which is an essential mechanism for the occurrence of osteolysis.

#### 4.1.4. Exosomes Prevent Excessive Osteolysis

Exosomes from mature osteoclasts can inhibit osteoclast formation through a paracrine mechanism [93, 94]. Exosomes from plasma of rheumatoid arthritis (RA) patients are similar to those in normal human plasma and significantly inhibit osteoclast production [95]. This inhibitory effect may be due to the role of the receptor RANK in mature osteoclast-derived exosomes as a decoy receptor that competitively binds RANKL similar to OPG. Further analysis showed that RANK levels in plasma exosomes are higher in RA patients than in normal subjects. This finding may be due to the increased production of mature osteoblasts. As such, osteoclast-derived exosomes may have a role in preventing excessive osteolysis persisting in inflammatory bone diseases. This process may involve a negative feedback regulation by the body to maintain the balance of bone metabolism and prevent excessive osteolysis. In another study, TNF-*α* pretreated MSCs secreted miR-1260b-containing exosomes in large quantities [62]. Exosomes containing miR-1260b target and block the Wnt5a-mediated RANKL pathway and inhibit osteoclast activity. MSC-derived exosomes have inhibitory effects not only on inflammation but also on osteoclast maturation. MSC-derived exosomes might be an excellent therapeutic direction for inflammatory bone diseases.

### 4.2. Exosomes and Bone Formation

Bone metabolism is strictly regulated by a balance of bone formation by osteoblasts and bone resorption by osteoclasts. Bone loss may be associated with increased osteoclast activity, reduced osteoblast activity, or a combination of both. Increased osteoclastic activity and decreased osteogenic activity play a role in inflammatory bone diseases. Osteoblasts, derived by direct differentiation of bone marrow mesenchymal stem cells, are responsible for bone formation in bone remodeling in vivo. Runt-related transcription factor-2 (Runx2) and osterix (OSX) are specific transcription factors for all osteoblast proliferation and differentiation stages, facilitating skeletal formation by transactivating bone matrix protein genes, including collagen type I, osteocalcin, and osteopontin [96, 97]. Exosomes in aseptic bone inflammation can affect osteoblast differentiation and activity in multiple ways by acting directly or indirectly on the Wnt signaling pathway or the expression of the transcription factors Runx2 and OSX (Figure 4).

#### 4.2.1. Exosomes Directly Affect the Activity of Osteoblasts

In aseptic inflammation of the bone, exosomes can directly influence the differentiation of osteoblasts, in addition to influencing osteoblast formation through inflammatory factors. Macrophage-derived exosomes are the leading force in inhibiting osteoblast differentiation in inflammatory bone diseases. miR-155 is enriched in M1 macrophage-derived exosomes [98]. miR-155 significantly decreases the expression of BMP2, BMP9, and Runx2, thus inhibiting osteogenic differentiation of MSC. miR-23a-5p-containing exosomes induced by RANKL are highly expressed in RAW 264.7 cells [99]. miR-23a-5p-containing exosomes effectively inhibit Runx2 and promote Yes-associated protein-1- (YAP1-) mediated MT1DP by suppressing osteoblast differentiation. Exosomes produced by RAW 264.7 cells after titanium particle treatment inhibit the differentiation of MC3T3-E1 cells [100]. The analysis of differentially expressed lncRNAs in exosomes produced by RAW 264.7 cells revealed that lncRNA NONMMUT000375.2 and lncRNA NONMMUT071578.2 might play an essential role in inhibiting osteoblast differentiation. However, no relevant experiments have explored the mechanism of action of these two lncRNAs involved in regulating osteoblast differentiation.

In addition, exosomes in the serum of patients with aseptic bone inflammation may also have remarkable effects on the differentiation of osteoblasts. In serum samples from patients with osteoporosis and ovarian denuded mice, the levels of exosomal miRNA were significantly higher than normal reference values [101]. Exosomes derived from osteoclasts containing miRNA-214 are delivered to osteoblasts through the ephrinA2-EphA2 signaling pathway and negatively regulate ATF4, thereby inhibiting osteogenic activity [102]. ATF4 is a crucial regulator of bone formation and determines the initiation and terminal differentiation of osteoblasts by transactivating the osteocalcin (OCN) gene and promoting the expression of other osteogenic genes, such as bone sialoprotein (BSP) and OSX [103]. In addition, lncRNA Hotair is classified as an essential regulator and is highly expressed in serum, which makes it a potential factor for the diagnosis of rheumatoid arthritis by serum assays [18]. Recent studies suggest that the mechanism of action of lncRNA Hotair may be related to the inhibition of osteogenic differentiation of MSCs by downregulating the expression of proteins related to the Wnt/*β*-catenin pathway [104].

#### 4.2.2. Exosomes Indirectly Affect Osteoblasts

The interaction of exosomes with inflammatory factors is a force to be reckoned with in inflammatory bone diseases. Exosomes promote the expression of inflammatory factors, such as TNF-*α* in inflammatory bone diseases, through various mechanisms, and these inflammatory factors inhibit osteoblast differentiation through various ways. TNF-*α* is one of the most potent inhibitors of osteogenic differentiation [105]. TNF-*α* independently inhibits the expression of procollagen *α*1 mRNA, resulting in reduced type I collagen synthesis that is a significant component of the mineralized bone matrix [106]. TNF-*α* can also induce the production of Dickkopf-1 (DDK1) and sclerotin (SOST), inhibitors of Wnt signaling, to inhibit osteoblast differentiation [107]. In addition, TNF-*α* can upregulate E3 ubiquitination ligase, which mediates the ubiquitination and degradation of Runx2, a key transcription factor for osteoblast differentiation [108–110]. Activation of NF-*κ*B also inhibits osteoblast production. The activation of NF-*κ*B upregulates miRNA-150-3p, inhibiting osteogenesis of mesenchymal stem cells by encouraging *β*-catenin degradation [111]. Besides, NF-*κ*B has a direct role in inhibiting BMP and Wnt signaling and negatively regulates bone mass through sclerostin [112]. Exosomes that activate inflammatory cytokines ultimately promote inflammatory bone diseases by promoting osteoclast formation and inhibiting osteoblast formation.

#### 4.2.3. Exosomes Prevent Excessive Reduction in Osteoblast Activity

While exosomes inhibit osteoblast activity in inflammatory bone diseases, exosomes that promote osteoblast activity are also produced due to the self-protection of the organism. One well-known example is that osteoclasts produce exosomes that promote osteoblast formation. Osteoclasts release RANK-containing exosomes that bind to RANKL on osteoblasts and stimulate RANKL to reverse signaling to promote osteoblast differentiation and bone formation via Runx2 [113]. Marton et al. showed higher levels of RANK in exosomes from patients with rheumatoid arthritis than in normal individuals [95]. However, whether this mechanism is self-protective and promotes osteoblast differentiation in aseptic inflammation of bone is unknown. Whether the reverse signaling of RANK-activated osteoblasts in exosomes plays a role in various bone metabolic diseases should be further investigated. Another important mechanism is that TNF, whose expression is facilitated by exosomes, can induce NFATc1 and promote bone formation [114]. Many experiments have observed a paradoxical role of NFATc1 in bone formation. It is unclear whether the dysregulation of bone formation in inflammatory bone disease is a coupled effect of increased bone loss leading to the increased bone formation or whether inflammation directly induces bone formation. Besides, exosomes containing miR-29b are highly expressed in TNF-*α*-treated RAW 264.7 cells. miR-29b may be associated with the regulation of osteogenic and osteolytic differentiation in aseptic inflammation of the bone [115]. Recent studies found that first miR-29b can promote proliferation and migration of rat bone marrow MSCs through PI3K/AKT and TGF-*β*/Smad signaling pathways [116]. These protective effects seen in inflammatory bone diseases may be related to the osteoblast-osteoclast dynamic balance, but further research is needed to elucidate the exact mechanisms.

## 5. Exosomes, Inflammation, and Bone Metabolism

Inflammation has the physiological purpose of restoring tissue homeostasis. However, uncontrolled or unresolved inflammation can lead to tissue damage, resulting in a variety of diseases characterized by a chronic inflammatory state [117]. Indeed, systemic inflammatory pathways are an essential component in the pathogenesis of inflammatory bone diseases. Inflammatory changes in the bone microenvironment can lead to excessive bone loss and altered bone formation. Inflammatory processes are associated with altered systemic bone remodeling, increased bone resorption, and impaired bone formation, and inflammatory mediators affect the differentiation and activity of osteoclasts and osteoblasts. Proinflammatory cytokines can enhance osteoclastogenesis and osteoclast activity. A decrease in bone-forming cell activity is also observed during the inflammatory process. The use of anti-inflammatory drugs (including glucocorticoids) can protect bones from inflammation-induced bone fragility. The inflammatory response occurs as an etiology of the disruption of the balance of bone metabolism. Exosomes appear to play a critical role in multiple signaling cascade responses in the inflammatory process because of their ability to carry inflammatory regulators, such as miRNAs and proteins, that can act on proximal and distant target tissues. Exosomes indirectly affect the activity of osteoblasts and osteoclasts by modulating the inflammatory response, thereby disrupting bone metabolic homeostasis. The loss of bone metabolic balance causes a range of symptoms, including inflammatory osteolysis and osteoporosis.

Homeostasis in bone metabolism is determined by the delicate balance between bone resorption by osteoclasts and bone formation by osteoblasts. This balance can be maintained between osteoblasts and osteoclasts through a variety of signaling pathways, such as RANKL/RANK, Ephrin/Eph, Wnt, complement, and TGF coupled together. Both osteoblast- and osteoclast-derived exosomes are involved in the coupling effect [118]. In an inflammatory environment, altered exosome expression can affect the coupling between osteoblasts and osteoclasts, thereby affecting the homeostasis of bone metabolism. Osteoclast-derived coupling factor, an exosome containing miR-214-3p, is altered in inflammatory bone disease, thereby affecting normal bone metabolism. As a coupling factor secreted by osteoblasts, miR-503-3p-containing exosomes can inhibit osteoclast differentiation. miR-677-3p, miR-680, miR-3084-3p, and miR-5000 are highly expressed in exosomes derived from mineralized osteoblasts. Let-7 is found in exosomes derived from osteoblast precursors and mature osteoblasts and can enhance osteogenesis by regulating the high mobility groups AT-hook 2 (HMGA2) and Axin 2. Osteoblast-derived exosomes containing miR-30d-5p, miR-140-3p of miR-133b-3p, miR-335-3p, miR-378b, and miR-677-3p also act as coupling factors that regulate osteoblast differentiation by autocrine means [119]. However, the role of exosomes and their level changes in bone homeostasis as osteoblast-osteoclast coupling factors in inflammatory bone diseases have not been well studied.

Overall, in inflammatory bone diseases, oxidative stressors can induce specific exosomal changes that aid in the inflammatory response. The inflammatory response subsequently affects the activity of osteoclasts and osteoblasts through the secretion of inflammatory factors or exosomes. It seems that the creation of an inflammatory microenvironment results in corresponding changes in exosomes, which are coupling factors in normal bone homeostasis, causing disturbances in bone metabolism. However, it is unclear whether these changes in the exosomes of osteoblast-osteoclast communication are caused by inflammation per se or by feedback changes following disturbances in bone metabolism. Finally, disturbances in bone metabolism in response to inflammation lead to increased bone loss and ultimately to inflammatory bone disease.

## 6. Clinical Application of Exosomes in Inflammatory Bone Diseases

One potential application of exosomes in inflammatory bone diseases is their use as a diagnostic and prognostic biomarker. The cargo in exosomes is highly dependent on the state of the releasing cell and its microenvironment. Thus, any pathological changes in the tissue microenvironment are reflected in the cargo content of the exosomes they release. Healthy subjects and patients with aseptic bone inflammation release exosomes containing varying concentrations of proteins, RNA, and other components into the circulation, which can be measured as biomarkers. Exosomes are widely available in a variety of body fluids and can be readily accessed. The exosomes encase the cargo and maintain its stability outside the cell. Techniques, such as reverse transcription-quantitative PCR, allow sensitive and specific detection of biomarkers, such as miRNAs in plasma and other body fluids. However, the technique of exosome purification still has many shortcomings. For example, as the most widely used method for the isolation of exosomes, differential centrifugation suffers from many disadvantages, such as coseparation of nonexosomal impurities, low reproducibility, low RNA yield, potential damage to exosomes, and low sample utilization [120]. Several studies have collectively shown differences in the fractions of exosomes extracted by different extraction methods [121–123]. The actual exosome content must be carefully differentiated by proper separation methods to prevent errors due to the cargo from other body fluid sources. In the future, if exosomes are used in clinical diagnostics, the method of exosome isolation must be improved to ensure reliable and reproducible results. Although few of these exosomal biomarkers have been documented to date, these exosomal components have considerable potential as diagnostic tools.

Exosomes of different origins and containing different components may exhibit inflammatory inhibition or osteolysis inhibition, making them potential tools for the treatment of inflammatory bone diseases. As natural endogenous nanovesicles, exosomes have various advantages, such as low immunogenicity, nontoxicity, and higher stability than other synthetic nanoparticles. The use of exosomes as an alternative to cellular therapies may be more straightforward, safer, and less costly, avoiding many of the problems associated with parental cellular drug delivery. In addition, exosomes can cross a variety of tissue barriers, enhancing the therapeutic effect of the adulterated molecules on target cells. Exosomes are used for three primary purposes in the treatment of inflammatory bone diseases: to modulate the immune response, to inhibit bone resorption and initiate bone repair, or to act as a carrier for therapeutic agents.

A massive example of modulating the immune response is the use of MSC-derived exosomes to suppress the inflammatory response. This method has been attempted in several experiments with promising results [124–128]. MSC-derived exosomes can ameliorate IL-1*β*-induced inflammatory effects and reduce apoptosis and matrix degradation during repair, as well as influence the conversion of macrophages to the M2 phenotype and participate in anti-inflammatory and regenerative responses. MSC exosomes may exert anti-inflammatory effects through specific miRNAs (miRNA-135b, miRNA-140-5p, miRNA21, miRNA-146a, and miRNA-181c), reversing the pathological inflammatory state without causing further apparent toxicity [129]. In a rat model, miRNA-135b in MSC-derived exosomes could promote cartilage repair by regulating TGF-*β*. Overexpression of miRNA-140-5p by exosomes derived from human synovial mesenchymal stem cells promoted cartilage tissue regeneration and blocked the side effects of OA [130]. The maturation mechanisms of miRNAs may vary depending on the cell type and cellular microenvironment. Mature MSC-derived exosomes contain more mature miRNAs than immature MSC-derived exosomes, and these miRNAs can promote chondrocyte proliferation, reduce apoptosis, and regulate immune responses [131]. Macrophage-derived exosomes may also contribute to the control of inflammation [132, 133]. The mechanisms through which these exosomes control aseptic inflammation should be further investigated. Further in vivo and clinical trials are needed to confirm its efficacy due to differences in vitro and in vivo and between organisms.

Osteoclast differentiation and function are responsible for inflammatory bone disease, accelerated by the control of cytokines produced in the inflammatory environment. The promotion of bone repair is another new target for the use of exosomes in the treatment of inflammatory bone diseases. For example, RANK-rich exosomes that inhibit osteoclast formation and promote osteoblast activity through reverse signaling can be used. However, better therapeutic outcomes may be achieved when treatment strategies that promote bone repair are used in conjunction with those that inhibit inflammation. Of course, exosomes also have a very high potential for drug delivery systems. Of particular interest is the macrophage-derived exosome expressing CD47, a surface signaling molecule used to evade immune surveillance. CD47 on the exosome membrane prevents endocytosis of exosomes by monocytes and macrophages, while CD9 and CD81 on the exosome surface promote the phagocytosis of exosomes. Macrophage-derived exosomes are therefore very attractive as drug delivery vehicles for the treatment of inflammatory bone diseases. Using these phagocytic properties, we can deliver drugs to target cells more efficiently. However, no studies have been conducted to prove whether such exosomes can be used to deliver anti-inflammatory drugs to reduce inflammatory diseases. Moreover, despite the efforts that have been made in these directions, substantial obstacles remain in obtaining exosomes with the desired properties.

## 7. Summary and Prospect

Exosomes have multiple functions similar to those of mother cells and have received increasing attention due to their natural portability and unique effects on target cells. With further research, we find that exosomes are closely associated with the pathological process of aseptic bone inflammation. Exosomes affect macrophage polarization and regulate the inflammatory response mainly through the NF-*κ*B signaling pathway. Alterations in inflammatory cytokines and exosome secretion caused by inflammation further affect bone metabolic homeostasis. These signals promote osteoclast differentiation via the RANKL pathway and inhibit the osteoblast activity via the Wnt pathway and the transcription factor Runx2, causing inflammatory osteolysis and promoting the development and progression of inflammatory bone disease. However, the body also produces exosomes that have a protective effect against the disease process. Exosomes have shown new pathogenesis in inflammatory bone diseases and provide a new direction for diagnosis and treatment. The use of exosomes has a very high potential in regulating inflammation and promoting bone repair. Reprogrammed or redesigned exosomes for disease treatment are promising in the future. However, the low yield and limited function of exosomes produced by current conventional methods essentially limit their further clinical application. Thus, further research on the biological properties of exosomes is urgently needed to improve the yields or enable the better function of exosomes. Overall, exosomes play an essential role in inflammatory bone diseases and are a promising therapeutic target.

## Figures and Tables

**Figure 1:** Process of exosome production and delivery. The plasma membrane internalizes to form early endosomes and gradually forms late endosomes. With the entry of intracytoplasmic proteins, lipids, DNA, and RNA cargoes, late endosomes produce a large number of intraluminal vesicles (ILV) inside the endosome, which gradually evolve into multivesicular bodies (MVBs). MVB can be degraded by the action of lysosomes to form lysosomes or fuse with the plasma membrane to release ILV further outside the cell to form exosomes. Exosomes released into the extracellular compartment enter the recipient cell in three ways: receptor-ligand binding, membrane fusion, and phagocytosis.

**Figure 2:** Effect of exosomes on macrophage differentiation. Toll-like receptor recruitment MyD88 mediates the activation of TNF receptor-associated factor-6 (TRAF6). TRAF6 promotes AP-1 signaling or NF-*κ*B activity via the I*κ*B kinase (IKK) complex. The IKK complex mediates the phosphorylation and subsequent degradation of I*κ*B*α*, while the IKK*α* dimer mediates the phosphorylation and degradation of p100, both of which can produce active NF-*κ*B. Exosomes containing oxidized phospholipids activate Toll-like receptors and promote the production of active NF-*κ*B. Inflammatory cytokines in exosomes bind to cytokine receptors, triggering the classical NF-*κ*B pathway, activating TAK1, and inducing NF-*κ*B activity. Exosomes containing miR-106b or lncRNA Hotair and those that are mesenchymal stem cell (MSC) derived promote I*κ*B*α* phosphorylation. Exosomes containing miR-223 inhibit the phosphorylation of p100 by IKK*α*.

**Figure 3:** Effect of exosomes on osteoclasts. The stimulation of RANK by RANKL initiates a long series of downstream signaling and gene expression cascades. Exosomes with proinflammatory effects increase the expression of inflammatory cytokines TNF-*α* and IL-1, which promote the expression of RANKL and enhance the sensitivity of osteoclasts to RANKL. IL-1 can also promote osteoclast maturation directly through MITF. Exosomes containing miR-214 or miR-106b promote osteoblast maturation by blocking the inhibitory effect of PTEN on the PI3K-Akt signaling pathway. RANKL-containing exosomes bind directly to RANK on the surface of osteoclasts and activate the RANK signaling pathway. By contrast, miR-1260b-containing exosomes inhibit the activation of Jun-N terminal kinase (JNK) by Wnt5a to suppress RANKL signaling. Mature osteoblast-derived RANK-containing exosomes inhibit RANKL signaling by competitively binding to RANKL.

**Figure 4:** Process through which exosomes affect osteoblasts. In the canonical pathway, Wnt signaling promotes *β*-catenin translocation to the nucleus, interacts with TCF/LEF, and stimulates the expression of downstream genes. Macrophage-derived exosome-induced inflammatory cytokines promote SOST expression, and the molecular chaperone LRP4 presents sclerostin to the Wnt coreceptors LRP5/6, thereby promoting inhibition of Wnt/*β*-catenin signaling by sclerostin. NF-*κ*B inhibits the degradation of *β*-catenin via miR-150-3p. TNF-*α* represses the expression of transcription factor Runx2 via E3 ubiquitination ligase. lncRNA Hotair inhibits the nuclear localization of TCF/LEF and *β*-catenin, thereby suppressing Wnt signaling. miR-155 and miR-23a-5p in exosomes directly repress Runx2 expression, while miR-214 represses activating transcription factor-4 (ATF4) expression. RANK signaling in exosomes triggers RANKL reverse signaling and promotes Runx2 expression.

## Abbreviations

TNF-*α*: Tumor necrosis factor-*α*
IL: Interleukin
PGE2: Prostaglandin E2
NF-*κ*B: Nuclear factor-kappaB
HMGB1: High mobility group box one
ILV: Intraluminal vesicles
MVB: Multivesicular body
EV: Extracellular vesicle
TLR: Toll-like receptor
LPS: Lipopolysaccharide
IFN-*γ*: Interferon *γ*
IRAK: Interleukin-1 receptor-associated kinase
TRAF: TNF receptor-associated factor
IKK: I*κ*B kinase complex
NIK: NF-*κ*B-inducing kinase
TAK1: Transforming growth factor *β*-activated kinase-1
MAPK: Mitogen-activated protein kinase
AP-1: Activator protein-1
MSC: Mesenchymal stem cell
MCP-1: Monocyte chemoattractant protein-1
CCL: Chemokine ligand
MIP: Macrophage inflammatory protein
PMMA: Polymethylacrylate
RANKL: Receptor activator of nuclear factor-kappaB ligand
VEGF: Vascular endothelial growth factor
MMP: Matrix metalloproteinase
iNOS: Inducible nitric oxide synthase
PTEN: Phosphatase and tensin homolog
CCR: Chemokine receptor
TRAP: Tartrate-resistant acid phosphatase
ERK: Extracellular signal-regulated kinase
JNK: Jun N-terminal kinase
NFATc1: Nuclear factor of activated T cell, cytoplasmic 1
MITF: Microphthalmia transcription factor
Akt: Serine/threonine protein kinase
PI3K: Phosphatidylinositol 3-kinase
ATF: Activating transcription factor
RANK: Receptor activator of nuclear factor-kappaB
GSK-3*β*: Glycogen synthase kinase 3*β*
SOST: Sclerotin
DKK1: Dickkopf-1
Runx2: Runt-related transcription factor-2
YAP: Yes-associated protein
OCN: Osteocalcin
BSP: Bone sialoprotein
OSX: Osterix
HMGA2: High mobility groups AT-hook 2.
